# Analysis of the Relationship between the Expression Level of TTR and APOH and Prognosis in Patients with Colorectal Cancer Metastasis Based on Bioinformatics

**DOI:** 10.1155/2022/1121312

**Published:** 2022-09-02

**Authors:** Ye Lu, Ying Wang, Yusong Qiu, Wenjuan Xuan

**Affiliations:** ^1^Hefei Cancer Hospital, Chinese Academy of Sciences, Hefei 230000, China; ^2^The First Clinical College, Xuzhou Medical University, Xuzhou 221004, China; ^3^Liaoning Cancer Hospital, Shenyang 110042, China

## Abstract

The expression of TTR and apolipoprotein H (APOH) genes and their relationship with prognosis in patients with colorectal cancer (CRC) metastasis by using bioinformatics analysis techniques are explored. The expression profiles of related genes in patients with CRC metastasis are retrieved from the Gene Expression Omnibus (GEO) database. The core genes transthyretin (TTR) and APOH are screened by constructing protein-protein interaction (PPI) network, and the corresponding patient data of 327 patients are extracted and included in the metastasis group. The TTR and APOH genes of 300 patients without CRC metastasis are screened and included in the control group. The relationship between the expression levels of TTR and APOH and the clinicopathological parameters of patients with CRC metastasis is analyzed. Kaplan–Meier survival curve is drawn to observe the influence of overexpression and low expression of TTR and APOH on the prognosis and survival of patients in the metastatic group. Receiver operating characteristic (ROC) curve is drawn to observe the prognostic efficacy of combined TTR and APOH detection in patients with CRC metastasis. The experimental results show that bioassay can confirm the close relationship between TTR, APOH, and patients with CRC metastasis. Regular detection of serum TTR and APOH expression can effectively assess the patient's condition and take measures to improve the prognosis of the patients.

## 1. Introduction

Colorectal cancer (CRC) is a kind of gastrointestinal malignancy with high mortality in clinical practice. With the development of national economy and society, dietary habits and structure gradually change, and the incidence of CRC is increasing year by year [1]. According to incomplete data, the number of colorectal cancer cases detected every year is about 1.25 million, and the mortality rate accounts for about half of the number of confirmed cases. The clinical features of early colorectal cancer are not significant, but more nonspecific, such as diarrhea and constipation. Therefore, most colorectal cancer patients can slow down the disease progression through surgery, chemotherapy, and other methods when they are diagnosed with end-stage cancer. However, uncontrolled tumor cell proliferation and metastasis are still important factors leading to high mortality of CRC [2, 3]. However, in recent years, with the continuous development of targeted molecular drug therapy, CRC patients can significantly prolong their prognostic survival by using targeted drugs, and the incidence of adverse reactions has been significantly improved, which greatly improves the quality of life of cancer patients [4]. Therefore, it is suggested that searching for related genes closely associated with CRC metastasis is of great significance in the diagnosis and treatment of patients and can also provide new therapeutic targets for the treatment of the patients with CRC metastasis [5]. As one of the largest gene chip databases in the world, Gene Expression Omnibus (GEO) database stores and accumulates a large number of PPIN data to construct the gene regulation network of tumor diseases [6, 7]. Above all, this study screened genes closely associated with CRC metastasis through GEO database and protein-protein interaction (PPI) network and further analyzed their expression in patients with CRC metastasis and prognostic value.

The rest of this paper is organized as follows.  Section 2 discusses related work, followed by data selection and the proposed methods designed in Section 3.  Section 4 shows the experimental results and analysis, and Section 5 summarizes the result of theoretical and empirical analysis and puts forward the direction of the future research.

## 2. Related Work

According to global incomplete data statistics, CRC, as the cancer disease with the second highest mortality and morbidity in the United States, has been on the rise year by year in China, and distant metastasis of tumor is the main risk factor for most patients with poor prognosis [8, 9]. According to relevant studies, among patients with CRC metastasis, about 30% of tumor cells have liver metastasis, and about 14% of patients still have liver metastasis after chemotherapy, which suggested that distant tumor metastasis was the main reason for poor prognosis of CRC patients [10]. Studies by many scholars on multi-step analysis of carcinogenic models have shown that somatic mutations give colon cells their respective growth advantages, thus accelerating the proliferation rate of tumor cells, which leads to distant metastasis of CRC tumors and initiation of invasive cancers [11]. Ongoing basic studies have suggested that oncogenes such as Ras and Myc and tumor suppressors such as P53 play an important role in the progression of CRC. Although the above basic studies can explain the pathogenesis of CRC to a certain extent, there is still no unified conclusion on the specific pathogenesis of CRC in clinical practice [12]. Therefore, constantly searching for new tumor markers and target genes is of great significance for predicting CRC metastasis and prognosis. In this study, GEO database was used to analyze the gene profiles related to CRC metastasis, and 95 DEGs with intersection were screened. TTR and APOH, whose expression is most closely related to CRC metastasis, were selected as research objects by constructing PPI network.

As a tetramer composed of four identical subunits, TTR can participate in the transport process of thyroxine, retinol, and other factors in the body through its identity as a transporter. In addition, when the body is under stress, albumin synthesis decreases rapidly, and the detectable TTR level in serum also decreases. It is suggested that TTR can reflect stress and albumin synthesis in the body to a certain extent [13, 14]. In addition, TTR, as a stable protein, is evenly distributed in human plasma and cerebrospinal fluid in normal body environment. When the balance of the body environment is destroyed, TTR is decomposed into monomers, resulting in a decrease in its expression level, which is consistent with the results in this study that TTR level in the patients with CRC metastasis is significantly lower than that in patients without CRC metastasis [15]. Wang et al. [16] indicated in the study that TTR can be synthesized by liver and choroid plexus and play an important role in cancer suppression in CRC, which can be used as a marker for early diagnosis of CRC and prognosis assessment, but its specific mechanism was not studied in depth. In addition, this study also showed that TTR was closely related to CRC stage and tumor size. It further demonstrated that TTR can be used as an indicator to evaluate the occurrence and prognosis of CRC and has high application value [17–19].

As a lipophilic protein molecule in human body, APOH can bind with lipopolysaccharide and activate NF-KB based on TLR4 pathway, thus further affecting the metastasis and invasion of tumor cells [20–24]. Guo et al. [25] pointed out that APOH can promote the differentiation of hepatocellular carcinoma cells and promote the progression of hepatocellular carcinoma. In this study, the expression of APOH in the patients with CRC metastasis was significantly higher than that in the patients without CRC metastasis. In addition, the patients with higher APOH expression level also have a decreased prognosis and survival rate, and it further suggested that APOH can play an important role in CRC metastasis [26].

Since both TTR and APOH have specific manifestations in the patients with CRC metastasis, this study observed the predictive value of enterprise combined detection on CRC metastasis by drawing ROC curve. ROC results showed that TTR combined with APOH had good predictive ability in evaluating the prognosis of the patients with CRC metastasis. Therefore, in the process of clinical treatment of such patients, the disease progression can be mastered through regular detection of serum TTR and APOH expressions, and the patients with specific manifestations of the above indicators can be closely monitored to timely take relevant measures to improve the prognosis of CRC patients [27].

## 3. Data Selection and the Proposed Methods

### 3.1. Data Selection

Related gene expression profiles of the patients with CRC metastasis are searched in the GEO database. Core genes transthyretin (TTR) and apolipoprotein H (APOH) are screened by constructing PPI network, and corresponding patient data of 327 patients are extracted and included in the metastasis group. TTR and APOH genes of 300 patients without CRC metastasis are screened and included in the control group. The comparison of baseline data between the two groups is shown in Table 1 (*P* > 0.05).

Inclusion criteria are as follows: (1) gene expression in CRC metastatic tissues and primary tissues and (2) complete gene expression.

### 3.2. The Proposed Methods

The gene profile data related to CRC metastasis are analyzed by GEO database, and the genes with significant expression difference between primary tumor and metastatic tumor (DEGs) are screened and further analyzed (*P* < 0.05). STRING and Cytoscape software are used to construct the protein network diagram of the protein encoded by DEGs, and the key genes are screened by MCODE.

After processing the data of GSE68468 and GSE81558 by GEO, 304 and 396 DEGs are screened out, respectively. A total of 95 DEGs with intersection of the two datasets are selected. Figures 1 and 2, respectively, represent the number of upregulated gene expression and downregulated gene expression in the two datasets, and the intersection part in red represents the common DEG part in the two datasets.

STRING and Cytoscape software are used to construct the protein network diagram of the protein encoded by DEGs, and MCODE is used to screen the key genes. The key gene screening is shown in Figure 3. The *P* values of the correlation between the key genes and the degree of CRC metastasis are shown in Table 2, and the two genes with the lowest *P* values are selected as the key genes of this study.

### 3.3. Statistical Treatment

All data in the study are collected and put into SPSS 25.0 statistical software for data analysis. (1) Measurement data: normality test is performed on the data first. If the data followed normal distribution and homogeneity of variance, they are represented by $\left(\bar{x}\pm s\right)$. Paired sample *T* test is used to test within the group, and variance comparison is used between groups. (2) Count data: descriptive statistical analysis is conducted by percentage, and *x*^*2*^ test is performed. (3) Survival analysis: Kaplan–Meier survival curve is drawn for the prognosis and survival of patients in the two groups. (4) PPI curve is used to observe the prognostic efficacy of TTR combined with APOH in the patients with CRC metastasis. *P* < 0.05 indicates significant difference.

## 4. Experimental Results and Analysis

### 4.1. Comparison of TTR and APOH Expression

Table 3 shows the comparison of the expression of TTR and APOH between the transfer group and the control group. It can be observed from Table 3 that compared with the patients without tumor metastasis, the expression of TTR in the metastatic group is significantly decreased, but APOH is significantly increased (*P* < 0.05).

### 4.2. Analysis of the Relationship between Different Expression Levels of TTR and APOH and Clinicopathological Parameters of CRC

The relationship between TTR expression and clinicopathological parameters of the patients with CRC metastasis is shown in Table 4. The regression forest plot of TTR and CRC clinicopathological parameters is shown in Figure 4. The relationship between APOH and clinicopathological parameters is shown in Table 5. The regression forest plot of APOH and CRC clinicopathological parameters is shown in Figure 5. It can be seen from the above experimental results that TTR and APOH are closely related to clinical stageand tumor size of the patients with CRC metastasis (*P* < 0.05).

### 4.3. Observation of the Influence of Overexpression and Low Expression of TTR and APOH

The influence of overexpression and underexpression of TTR on prognosis and survival of patients with CRC metastasis is shown in Figure 6, and the relationship between APOH expression and prognosis and survival is shown in Figure 7. Through the above experimental results, it can be observed that the prognosis and survival of patients with high TTR expression are significantly better than those with low expression, but the prognosis of patients with high APOH expression is worse than that of the low expression group (*x*^*2*^ = 1.274,1.763; *P* = 0.031,0.012).

### 4.4. Observation of the Prognostic Efficacy of Combined TTR and APOH Tests for the Patients with CRC Metastasis by ROC Curve

The diagnostic efficiency of each index is shown in Table 6. The prognostic curve of ROC for the patients with CRC metastasis is shown in Figure 8. Through the above experimental results, it can be observed that TTR combined with APOH has a high predictive efficacy for the prognosis of the patients with CRC metastasis.

## 5. Conclusions and Future Directions

The expression of TTR and APOH genes and their relationship with prognosis in patients with CRC metastasis by using bioinformatics analysis techniques are explored. TTR and APOH screened based on bioinformation technology are closely related to the patients with CRC metastasis, and they can be used as effective serum markers for the diagnosis of CRC and prognosis assessment. However, the specific mechanism between TTR, APOH, and CRC is not further analyzed in this paper, so there are still some deficiencies in this study. In the future, basic research can analyze its related mechanism of action, further elaborate the related mechanism of distant metastasis of CRC, and provide new potential targets for diagnosis and treatment of patients with CRC metastasis.

## Figures and Tables

**Figure 1:** Upregulated gene.

**Figure 2:** Downregulated gene.

**Figure 3:** Key gene screening.

**Figure 4:** Regression forest plot of TTR and CRC clinicopathological parameters.

**Figure 5:** Regression forest plot of APOH and CRC clinicopathological parameters.

**Figure 6:** Relationship between TTR expression and prognosis and survival.

**Figure 7:** Relationship between APOH expression and prognosis and survival.

**Figure 8:** Prognostic curve of ROC for the patients with CRC metastasis.

**Table 1:** The baseline data.

	Transfer group (*n* = 327)	Control group (*n* = 300)	*t/x* ^*2*^	*P*
Age (years)	43.21 ± 9.53	44.31 ± 9.31	−1.460	0.145

Gender			3.638	0.056
Male	198 (60.55%)	159 (53.00%)		
Female	129 (39.45%)	141 (47.00%)		

BMI (kg/m^2^)	23.35 ± 2.47	23.19 ± 2.43	0.817	0.414

Level of education			1.248	0.523
Primary and below	102 (31.19%)	87 (29.00%)		
Junior to senior high	159 (48.62%)	155 (51.67%)		
University and above	66 (20.18%)	58 (19.33%)		

**Table 2:** *P* values of key genes.

Gene	*P* value
APOH	3.09*E* − 09
HPD	2.18*E* − 05
HPX	3.58*E* − 06
C6	4.63*E* − 03
CFHR5	5.26*E* − 04
SLC2A2	3.63*E* − 05
ITIH1	5.32*E* − 03
CP	4.37*E* − 03
F9	3.59*E* − 05
TTR	4.65*E* − 08
AMBP	4.21*E* − 04
KING1	5.37*E* − 04
F2	4.19*E* − 05
CPB2	5.18*E* − 07
GC	4.74*E* − 04
HRG	4.04*E* − 05
AHSG	3.48*E* − 03
SERPING1	2.18*E* − 06

**Table 3:** Comparison of the expression of TTR and APOH between the transfer group and the control group.

Group	*n*	TTR mRNA	APOH mRNA
Transfer group	327	3.64 ± 1.02	5.42 ± 1.21
Control group	300	11.24 ± 3.22	9.56 ± 2.10
*T*		−40.525	−30.549
*P*		<0.001	<0.001

**Table 4:** The relationship between TTR and clinicopathological parameters.

	Number (*n* = 627)	High expression	Low expression	*x* ^*2*^	*P*
Gender				0.006	0.940
Male	357	169 (47.34%)	188 (52.66%)		
Female	270	127 (47.04%)	143 (52.96%)		

Age (years)				0.108	0.743
≥40	445	243 (54.61%)	202 (45.39%)		
<40	182	102 (56.04%)	80 (43.96%)		

TNM staging				341.369	<0.001
I ∼ II	300	257 (85.67%)	43 (14.33%)		
III ∼ IV	327	39 (11.93%)	288 (88.07%)		

Tumor diameter (cm)				241.158	<0.001
≥4	387	59 (15.25%)	328 (84.75%)		
<4	240	186 (77.50%)	54 (22.50%)		

**Table 5:** The relationship between APOH and clinicopathological parameters.

	Number (*n* = 327)	High expression	Low expression	*x* ^*2*^	*P*
Gender				0.556	0.456
Male	357	176 (49.30%)	181 (50.70%)		
Female	270	125 (46.30%)	145 (53.70%)		

Age (years)				0.593	0.441
≥40	445	227 (51.01%)	218 (48.99%)		
<40	182	99 (54.40%)	83 (45.60%)		

TNM staging				309.678	<0.001
I ∼ II	300	248 (82.67%)	52 (17.33%)		
III ∼ IV	327	41 (12.54%)	286 (87.46%)		

Tumor diameter (cm)				203.394	<0.001
≥4	387	71 (18.35%)	316 (81.65%)		
<4	240	182 (75.83%)	58 (24.17%)		

**Table 6:** Diagnostic efficiency of each index.

	95% CI	Sensitivity (%)	Specificity (%)	AUC	Cutoff value
The joint detection	0.861 ∼ 0.958	91.10	87.40	0.926	—
TTR	0.724 ∼ 0.896	78.50	72.40	0.804	4.29
APOH	0.712 ∼ 0.887	75.70	74.10	0.821	6.82

## Data Availability

The simulation experiment data used to support the findings of this study are available from the corresponding author upon request.
